This article has been retracted.

# Effect of Protein Nutrition Level on Protein Metabolism during Volleyball Exercise Based on Edge Computing in the Medical System

**DOI:** 10.1155/2022/1614748

**Published:** 2022-01-12

**Authors:** Jicheng Yang, Ning Du, Wei Jiang, Chenzhe Liu

**Affiliations:** ^1^Physical Education College, Jinan University, Guangzhou 510632, Guangdong, China; ^2^School of Physical Education, South China Normal University, Guangzhou 510006, China; ^3^Department of Sports Physiology, Beijing University of Physical Education, Beijing 100089, China

## Abstract

With the rapid development of the Internet of Things, 5G, and communication technologies, the growth of various types of data has shown an exponential trend. Edge computing technology provides users with almost unlimited computing power through a large number of high-performance servers in the data center. It is one of the important solutions for big data analysis and processing. Volleyball has caused a great wave in China as early as the 1960s, but people pay little attention to the physical quality of volleyball players. At the same time, in the medical field, it is difficult to give a clear value to the athlete's protein requirement. Therefore, this article aims to observe the specific values of protein metabolism in volleyball at different levels of protein nutrition. By designing controlled experiments, then these rats under three nutrient levels of protein were observed and protein metabolism was analyzed after volleyball. The results of the study show that volleyball exercise can reduce the nitrogen balance and gastrocnemius nitrogen content. The nitrogen balance of the 17% group decreased from 388 mg/day before exercise to 336 mg/day, and the gastrocnemius nitrogen content decreased by up to 5.2%; serum urea nitrogen concentration and liver nitrogen content are increased, indicating the enhancement of protein catabolism. Different protein nutrition levels have different effects on protein metabolism during volleyball. The protein intake level of 17% is more conducive to resist the protein decomposition caused by volleyball. It can be seen that, based on edge computing technology, the influence factors of protein nutrition level on protein metabolism during volleyball sports can be well explored, and the research results are also very valuable.

## 1. Introduction

Human life involves many elements, and protein is one of the important elements. The human body needs a certain amount of protein every day to maintain balance. Protein supplements athletes' energy, strengthens human muscles, promotes the normal synthesis of human hemoglobin, accelerates metabolism, and eliminates fatigue. It has important practical significance. During exercise, the speed of protein synthesis will be greatly reduced [1]. Exercise, especially strength exercise, can stimulate muscle protein synthesis, leading to increased lean body mass and muscle mass; in addition, hemolysis intensifies in the early stage of heavy-load training, prompting red blood cells to strengthen the synthesis of mitochondria and the synthesis of enzymes. Starting from volleyball, this article studies the effect of protein nutrition level on protein metabolism in a single sport, narrowing the research direction, making the entire research process more detailed and the research conclusions more authentic. Volleyball is one of the most popular sports in China. Men, women, young and old are happy to participate in it. Volleyball can improve people's physical quality and sports ability such as strength, speed, flexibility, endurance, bounce, and reaction and improve the functional status of various organs and systems of the body. Generally speaking, protein can provide 5.5% of the total calories consumed during exercise. However, further research is needed to determine the protein content required by the body during sports and the relationship between the protein metabolism level of volleyball players during sports and the protein nutrition level of the body. Current research techniques cannot directly explore the reasons for this [2].

In recent years, society has gradually entered the “big data” era, and the emergence of cloud computing has enabled the ability to process and use big data to increase day by day. Cloud computing has been vigorously promoted with its advantages of low operating costs, dynamic scalability, and simplified operation and maintenance, and cloud computing-related industries have developed rapidly in China. On this basis, the state put forward medical informatization as an important development direction of medical physique reform [3]. Although cloud computing has announced the possibility of providing computer services at a lower cost, it also allows hackers to invest less money and obtain huge network computing power. Hacker attacks will pose a serious threat to user data security. Therefore, before these security problems and risk factors are properly managed, cloud computing is difficult to be effectively utilized. The nearby intelligent services provided by edge computing technology can meet the key requirements of agile connection, real-time business, data optimization, application intelligence, security, and privacy protection. An intelligent, flexible, and elastic medical network is built at the edge of the network. At the same time, its extremely strong computing power can do a good job on this subject [4, 5].

In order to use the edge cloud computing technology in the medical system to study the subject, Zhang et al. aim to use the security relationship of data information in edge technology computing and the technical characteristics of data privacy information protection to study the protection methods of commercially confidential information. He proposed a theoretical system and technical architecture centered on the application of data security technology. Experimental data shows that identification errors mainly occur when identifying nonabnormal data as abnormal data. The analysis and identification of abnormal information data are basically accurate, and various processing tasks can be completed quickly, and the abnormal information data can be eliminated to meet the requirements. However, the research motivation is unclear [6]. Mitchell's research has shown that healthy individuals have a significantly constant skeletal muscle mass for most of their adult life, indicating the existence of homeostatic mechanisms. The amino acids consumed by dietary protein and the amino acids consumed by muscle protein synthesis are offset, making muscles exist in dynamic balance. The study uses atomic absorption spectroscopy, based on human studies, to describe the human bone protein metabolism in detail [7]. Ato proposed that the combination of exercise and nutritional intake can enhance protein anabolism more than exercise or nutritional intake alone. On this basis, the mechanism of protein anabolism based on the combination of exercise and nutritional intake was discussed, and recommendations were made to promote protein anabolism based on the latest research results. It is proposed that effective protein intake and functional food intake help to adapt to exercise to the maximum extent [8].

Compared with the previous studies on protein metabolism, the innovations of this paper are as follows: (1) the physiological function of the protein and the effect of endurance exercise on protein metabolism are analyzed in detail, which provides a comprehensive theoretical basis for the research. (2) The experiment was carried out in three batches to strictly control the experimental variables. The determination of serum urea nitrogen can also be used as a reliable chemical index to study the effects of different protein nutritional levels on protein metabolism in volleyball. (3) The third point is to use the nitrogen balance experiment method. The nitrogen balance experiment is an experiment to determine the protein demand of the human body, that is, to measure and compare the relationship between the intake of nitrogen and the discharge of nitrogen. It is difficult to directly measure the relationship between the protein content in the human body, and the change of nitrogen can reflect the protein metabolism. Combined with keas method, an experimental model of protein metabolism in Volleyball was established.

## 2. Introduction to Protein Nutrition Level Theory and Edge Computing

Protein is an important part of the human body. People need to consume a certain amount of protein every day to maintain the body's balance. It can be seen that human life is inseparable from protein, and protein itself is also a part of the important structure of normal human cells. Proteins have different structures and many physiological functions, mainly four functions [9].

One is the catalytic function. Chemical reactions need to occur in the body to provide nutrients to maintain the normal functions of the body and maintain its balance. Enzymes are catalysts for many chemical reactions [10]. Only in this way can a person's metabolism be more effectively and correctly controlled, and wastes from the body can be effectively discharged from the body as soon as possible. After a number of scientific experiments, protein coenzymes are the main components of more than 1,000 proteases in the human body [11]. Therefore, protein coenzymes have certain biocatalytic functions and are important substances for maintaining human body functions. Second is the transportation function. Human tissue is an organic whole, and various physiological digestive activities such as blood circulation and rapid oxygen delivery require organic carriers. Protein nutrition is an effective nutrient carrier that guarantees the maintenance of the normal physiological transportation of the human body, and an effective nutritional tool that promotes the maintenance of the normal physiological function of the human body. Therefore, the effective transportation of substances in the human body and the normal operation of human functions require proteins to complete the transportation activities and ensure its organic circulation. Third, motor function, as we all know, the human body mainly exercises through abdominal muscles. The main nutrient component of muscle is muscle protein, and the normal contraction and relaxation of human muscles are related to its protein content. The muscle development of ordinary football players is more developed than the abdomen and other muscles of many ordinary people. This is because ordinary athletes have a certain measurement standard for their daily eating habits, and they need to consume a lot of protein, fat, water, and other substances every day. It can be seen that protein is an indispensable and important factor in human exercise and has certain exercise functions. Fourth is the hormonal function. Hormones play a role in drug therapy. From a biological point of view, many hormones are mainly composed of proteins, so proteins have certain hormone functions. Protein and peptide metabolism hormones are mainly important metabolic hormones in various animals, which can be used to regulate and help control the normal physiological metabolic activities of various animals. For example, insulin polypeptide can effectively reduce human blood sugar; however, heme polypeptide is an active polypeptide with 29 main amino acid residues and a molecular weight of 3585. Its pharmacological effect is completely opposite to that of active insulin, which can promote glycogenolysis and gluconeogenesis and increase blood glucose concentration [12]. The hormones in people's lives are often exposed to the outside, but it will cause certain damage to the human body to minimize the use of hormones.

Protein nutrition level plays an important role in maintaining human body functions. Among them, the level of protein nutrition directly affects the human immune system. Protein deficiency not only affects the body's cellular immunity but also hinders humoral immunity. Protein can accelerate the proliferation of neutral lymphocytes, differentiate, and delay allergic reactions. When the human body protein content is insufficient, the chemical reaction inhibition ability of the antibody or antigen binding to it will decrease, and the complement concentration will also decrease. The synthesis of antibodies requires the participation of a series of proteases. The level of antibody levels of immune proteins in the body will directly affect the antibody content of various immune enzymes in human cells, thereby directly changing the rate of cell synthesis and differentiation of antibodies in the body and directly affecting the effect of cellular humoral immunity effect. The low content of protein cannot fully meet the basic needs of ensuring the normal maintenance of the body's immune system. Only when the protein and fat content in the daily life diet gradually reaches a certain balance level, the body's autoimmune system potential damage can gradually reach the best defense state. However, if the protein nutrition level is too high, it will also cause adverse effects on the human immune function, such as causing excessive body burden.

The body's requirements for protein nutrition level when participating in sports activities are different from our daily activities. The diet of athletes has scientific standards. There is a certain relationship between the protein nutrition level of athletes and sports events and their own body weight. For the same sport, there are protein intake standards for different genders, weights, and training intensity. Nutritionists need to reasonably arrange specific diets according to the actual nutritional status of all athletes to effectively promote the reasonable diet and healthy growth of all athletes. The results of the study show that the average daily protein requirement for long-term moderate and high-intensity weight-bearing exercise should be 2.5–3.0 g/kg, and the average daily protein requirement for speed and weight-bearing power athletes is 2.4–2.59 g/kg [13]. It is generally believed that when athletes are just beginning to perform strenuous exercise aerobic training because strenuous training is not fully adapted, the degree of damage to body cell function increases, and the metabolism of synthetic substances such as muscle collagen and red blood cell regeneration of the body is hyperactive. As well as the body's stress hormones and central nervous function regulation, other adverse reactions often lead to negative nitrogen balance and even cause severe exercise-induced anemia; strenuous exercise will also increase the amount of protein excreted in the urine. However, after a period of adaptation, the nitrogen balance will be improved. Therefore, in the early stage of strenuous exercise and when the exercise intensity is high, the protein nutrition level should be appropriately enhanced. According to the results of the nitrogen balance experiment, it is recommended that the daily protein intake of children participating in sports training should be between 2.0 g/kg and 3.0 g/kg. This is also a general standard, and different experts, scholars, and research data also have certain differences. Strictly speaking, every ball player will have his own special characteristics. Nutritionists should reasonably arrange the average intake of human protein according to the actual physical conditions of professional athletes and the actual working conditions in a timely manner to help ensure the normal sports training of professional athletes. This also promotes the continuous enhancement of professional trainers' performance.

Prolonged endurance exercise will increase protein metabolism, so protein nutrition levels will also increase. The increase in protein intake is also affected by glycogen storage. In endurance sports, when the concentration of muscle and glycogen is sufficient, the obvious increase in protein nutrition and energy consumption is limited to only 4% of the total human food nutrition and energy consumption. When the content of glycogen acid in a human body is completely exhausted, the loss can only increase downward by 10% at the same time. During long-term exercise (3.75 hours), the anaerobic energy consumption generated by the oxidation process of amino acids accounts for 4%–8% of the total oxidative energy consumption. Therefore, in addition to high-intensity endurance training, it is obviously reasonable to increase protein requirements by 10% [14]. Strength balance training also requires a slight increase in the total body protein and fat intake due to the increase in fat consumption of human muscles and soft tissues. The exercise intensity is high, the number of training sessions is large, and the protein metabolism is enhanced, which needs to be increased. In addition, for those professional ball players who need to strictly control their normal weight, they usually think that they should choose as many fish and meat as the main foods that are rich in protein, high in fat, and high in bone density to satisfy their demand. Protein foods can account for 18% of total calories. However, how the protein nutrition level affects the protein metabolism in volleyball and how much protein content is the most appropriate, these specific situations still need to be known according to the specific situation of volleyball players. Therefore, the level of protein nutrition depends on the situation.

In order to better study how protein nutrition level affects protein metabolism in volleyball, we established a nitrogen balance measurement model and designed a data analysis system based on edge calculation.

Nitrogen balance is the balance between nitrogen intake and production. The nitrogen balance test is a classic method for studying protein requirements, measuring daily nitrogen intake and nitrogen excretion, and comparing the ratio of the two. Its main applications include the overall balance of nitrogen, the positive balance of nitrogen, and the negative positive balance of nitrogen. Its general form is as follows:

(1) $$\begin{array}{c} \frac{\left[d-\left(n+f+p\right)\right]}{\sqrt{n^{2}+{\left(f-p\right)}^{2}}}=dt\;. \end{array}$$

Among them, *d* is the intake of nitrogen, and *n*, *f*, and *p* represent the emissions of carrying nitrogen. We need to use the keas method to determine the value of *N*, *F,* and *P*. The calculation formula of crude protein in the keas method is as follows:

(2) $$\begin{array}{c} X=\left(V1-V2\right)\times C\times 0.0140\times 6.25. \end{array}$$

Edge computing is a new ecological model. By converging five types of resources, including network, computing, storage, application, and intelligence, at the edge of the network, it can improve network service performance and open network control capabilities, thereby inspiring new models similar to the mobile Internet.

Edge computing was originally a key technology to solve the 5G network delay problem. In recent years, it has been tried to be used in emerging fields such as the Internet of Vehicles and the Internet of Things [15]. The abovementioned problems in the processing of cloud computing can be solved by edge computing technology. As a hot technology, edge computing has been widely used in the business field. Among them, Internet companies hope to extend their existing cloud service capabilities to edge networks with the help of their own relevant advantages in the service industry. Communication companies hope to use edge computing technology to further tap the value of network connection equipment and improve their technological status in the consumer Internet of Things and Industrial Internet by strengthening the relevant performance of the access side network. The approach of industrial enterprises is to combine IT and OT. That is, traditional enterprises use IT solutions in local cloud architecture and add industrial operation technology to GE or non-GE facilities. They hope to use the Industrial Internet as their main position, use their own industrial network connections and industrial Internet platform services to give full play to their advantages, and establish new business models [16].

On the basis of edge computing, it provides medical workers with a medical management system that supports hierarchical division, two-way referral, and provides data analysis services. The mobile medical information system integration platform is a medical data sharing platform designed for mobile terminals, primary medical care, and community family medical care based on the IHE (Integrating the Healthcare Enterprise) technical framework of medical information system integration. IHE is a technical framework designed to improve the sharing of information and data between medical systems. It specifically describes the information transmission between various systems based on the IHE system document standard. On this platform, the advantages of edge computing can be better utilized, and protein metabolism can be explored in depth from a clinical perspective.

## 3. Theory of Endurance Exercise and Protein Metabolism

In endurance exercise, most of the protein synthesis of muscle tissue is inhibited, but there is no instance in the exercise of muscle protein being broken down. Otherwise, it is not in it. On the one hand, the liver, muscle vasoconstrictor enzyme, and protein binding decomposition reaction speed varies. The speed of the synthetase slows down, the release of amino acids increases, and the amino acids in the metabolic pool increase; on the other hand, exercise will increase the alanine released by glucose, especially in this process (when the rate of alanine release 30 mol/L, moderate-intensity exercise to 70 mol/L, and vigorous exercise soaring to 170 mol/L) cycle in order to maintain blood sugar levels; during the recovery period after exercise, the exercise muscles produce methyl histamine cad, urine excretion increased, methyl histidine excretion increased, to provide evidence for conversion into muscle protein; exercise has a stable isotope tracing method, which can show exercise in the process of protein metabolism, so exercise has an effect on protein synthesis and decomposition has obvious effects [17].

Long-term endurance exercise consumes the sugar in the body. Due to the limited sugar reserves in the body, the glycosylation pathway of amino acids is activated. After removing amino acids, the carbon skeleton of most amino acids in the body can enter the triaxial cycle or anaerobic glycolysis metabolic pathway and can also be converted into glucose after oxidation to help maintain blood sugar [18]. Alanine and glutamine account for 30% of the amino acid. In the process of exercise metabolism in human muscles, acetylacetonate produced by the oxidation reaction of glucose reacts with other amino acids (such as lysine) to hydrolyze. Alanine can enter the human blood and directly return to the human liver. In the human liver, it directly generates a large amount of glucose through the pathway of gluconeogenic enzymes and metabolic enzymes, which greatly increases the main source of blood glucose metabolism in the blood of human exercise hypoxia. The biological oxidation process of glutamine glucose should also have a similar cyclic glutamine-glucosamine oxidation cycle, which is also related to the maintenance of blood sugar during exercise.

Generally, protein provides a small proportion of energy during exercise, accounting for about 5% to 7% of the total heat energy demand. In endurance exercise, the percentage of amino acid supply increases after muscle glycogen is depleted. In the process of alanine-hydroxy glucose and glutamine-hydroxy glucuronide cycle conversion, part of the hydroxy glucuronide produced by the enzymatic conversion process of alanine and glutamine in the liver can be reoxidized and enter the human muscles. Fat cells oxidize fat to produce more energy. During the oxidation of phenylalanine and glutamine produced by keto acids in human musculoskeletal tissues, an amino acid that provides this amino acid is converted into keto acid by invertase, which can enter into the synthesis of aerobic keto acid metabolism enzyme pathways to provide keto acid oxidase function. In addition, muscles use amino acids circulating in the blood. Some studies have shown that the muscle uptake rate of branched-chain amino acids increases during exercise, while long-term vigorous exercise can increase the amount of oxidation several times [19]. As mentioned above, the increase in alanine concentration during exercise is mainly due to the enhancement of protein metabolism during exercise, which makes the amino acids produced, especially branched-chain amino acids, easily converted into pyruvate under the catalysis of pyruvate and produce alanine. In the constant perfusion experiment of isotope 13C-labeled leucine, it was observed that the oxidation rate of leucine increased by 2 times after 50% intensity exercise for 2 hours, and the absolute value of leucine increase was equal to the requirement of 90 for the amino acid. Therefore, the powerful effect of supplementing branched-chain amino acids has attracted widespread attention. Although the use of branched-chain amino acids, in theory, can improve the energy supply of working muscles, so far, it has not been proven to improve performance in well-designed randomized controlled clinical trials.

As mentioned above, in the process of endurance exercise, the oxidative exercise effect of leucine is also greatly enhanced. However, whether it can increase the mutual oxidative combination of all two amino acids remains to be proved by experiments. The intermediate metabolism of certain important amino acids can produce tricarboxylic acids or cyclic metabolic catalyst products, which have a good regulatory effect on the human body's exercise metabolism process and the human muscle metabolism process. Because it greatly increases the active oxidation reaction capacity of the ethyl cycle to the formyl ethyl peptide cocoa produced by the reaction of glucosamine and other free amino fatty acids. In addition, the main metabolites of these major amino acids can also be converted into pyruvate by dodecyl phosphate pyruvate oxidative kinase and pyruvate oxidative kinase. The increase in pyruvate production can lead to an increase in amino acid oxidation during exercise. The oxidation of amino acids is an important process in the human body.

## 4. Establishment of an Experimental Model of the Protein Metabolism in Volleyball

### 4.1. Experimental Animals and Establishment of Model

The Zoology Center of the Medical Sciences provided 96 male Wistar rats weighing (69 ± 7) g. During the experiment, each rat was fed separately in a cage. Specially prepared feed was required during feeding, free drinking water, room temperature (25 ± 2) °C, and natural light.

#### 4.1.1. First Batch of Experiments

24 male Wistar rats are the only choice for introducing experimental animals, and in order to study the effect of different content of protein feed on energy supply in Wistar rats, they are randomly divided into 3 groups, namely, three different levels of protein intake groups (hereinafter referred to as each group is 7%, 17%, 27%), each grouped in eight cage methods, according to the main nutrient composition of the feed ain-76 animal species, as shown in Table 1.

The various nutrients in various types of feed animals mainly refer to the weight of various feed animals. The percentage of carbohydrates is also different. The energy provided by the three levels of protein accounted for 7.8%, 18.6%, and 29.9% of the total energy of the feed, respectively. Based on the average food of the rats with the least food intake as the standard, each group was given an equal weight of feed so that the energy intake of each rat was equal. After eating for 45 days, the rats were forced to play volleyball until they collapsed, and the fatigue time of each rat was recorded.

#### 4.1.2. The second Batch of Experiments

There are 24 male Wistar rats, and the animal source is the same as above. In order to study different levels of protein metabolism, they were randomly divided into 3 groups with 8 animals in each group. They were fed the above three protein levels separately and fed in a metabolic cage. The feeding method is the same as above. After the 3rd day, they were fed, urinated for 1 hour a day, exercised continuously for 5 days, and collected the daily urine and feces. During the urination period, feces were collected on the 3rd, 2, 4, and 6 days after urination. The keas method analyzes the nitrogen intake in urine, and the feces excrete nitrogen. Nitrogen balance is equal to nitrogen intake minus emissions.

#### 4.1.3. The Third Batch of Experiments

In order to study the effect of protein nutrition level on the nitrogen content of gastrocnemius muscle and liver, they were randomly divided into 6 groups, each with 8 animals, namely the control group and the experimental group with several protein intake levels. The control group did not play volleyball, and the feed formula and measurement method were the same as those mentioned above. After 45 days, the experimental group performed volleyball exercises for two hours at a temperature of (25 ± 2)°C. Immediately after exercise, they were killed by decapitation. Blood samples, insulin, and gastrocnemius muscle were taken at 3000 rpm/heart was separated for 15 minutes. They were stored in a low temperature environment. The serum urea concentration was determined by the diacetyl method, and the instrument was Shimadzu UN-120-20 spectrophotometer. The content of gastrocnemius muscle nitrogen and serum nitrogen is determined by the advanced keas method.

### 4.2. Observation Items and Methods

Every 5 days, the weight of the rats was measured by an accurate electronic balance, and the average body weight of rats with a protein level of 7%, a protein level of 17%, and a protein level of 27% was calculated, respectively. In the preexercise, mid-exercise, and postexercise periods, nitrogen intake, urine, and excrement are measured for nitrogen balance, and nitrogen balance is calculated. The urine and stool samples collected were analyzed for the last three consecutive days in the fourth week before exercise. Urine and stool samples collected on the third, fourth, and fifth days of the exercise were analyzed for urine and fecal nitrogen, respectively. Urine and stool samples were collected 2, 4, and 6 days after exercise, and the nitrogen in the urine and stool was analyzed daily. The nitrogen balance is determined by the kea's method. The serum urea nitrogen was determined by the diacetyl method. The automatic keas method was used to determine the content of amino acid carbon and nitrogen compounds in the gastrocnemius muscle and liver blood. Use automatic amino acid concentration analyzer to determine serum amino acids, use 5% of serum to combine with sulfosalicylic acid to precipitate protein, and the volume ratio of serum to the salicylic acid to precipitate protein is 1 : 1.5. After fully mixing with serum, put the instrument at −18°C and freeze for more than 30 minutes, and analyze the amino acid concentration of the supernatant. The amino acid condition of the instrument should be a physiological liquid column (4.0 mm∗150 mm), lithium salt buffer system, filler 2619f resin, 34∼ 68°C temperature gradient×4.

### 4.3. Western Blot Detection of Protein Metabolism

The extensor muscles of each test rat's limbs were taken out and stored frozen at −80°C and 50 mg, respectively. It was quickly extracted and put into a small tube containing polymerization inhibitor and lysate and washed for 20 s three times. Centrifuge the supernatant for 30 minutes. Using BCA to measure proteins and compounds, it can be directly used to accurately measure the average concentration of various proteins and compounds in all test samples when determining the measurement kit and adding the corresponding ratio of lysis substances and buffers. Adjust the concentration to the same level, and denature at 70°C for 10 minutes. SDS-PAGE gel electrophoresis at 200 V for 45 minutes. Prepare 5% skimmed milk to seal the PVDF membrane for 1 hour. Prepare with 5% BSA solution and incubate overnight on a shaker at 4°C. After washing the next day, incubate for 1 hour on a shaker at room temperature. After cleaning, put the adhesive strip into the chemiluminescence reagent imaging and development system, and add a chemiluminescence reagent meter on the adhesive strip to expose and develop the adhesive strip. Use Image Lab5.1 software to analyze the gray value of the fluorescent protein in the gel strip to accurately calculate the gray relative expression of the gel strip and the target protein [20]. Use SPSS to process the experimental data and describe the results in the form of mean ± standard deviation. A one-way variance test was used for comparison between groups.

## 5. Analysis of the Effect of Protein Nutrition Level on Protein Metabolism in Volleyball

### 5.1. Analysis of Three Protein Nutrition Levels on Rats' Body Weight Gain during Volleyball Sport

First, statistical analysis of the weight of experimental rats. Considering the influence of food on the weight of rats, the weight of rats was measured twice in the morning and evening. Therefore, the data in the figure is based on time and presents certain distribution characteristics. It was found that under the nutritional levels of the three proteins, there was no significant difference in the weight gain of rats. Although there was no significant difference in the nutritional levels of the three proteins in rats, the volleyball exercise time of the 7% group and the 17% group was 22% and 25% longer than that of the 27% group and 22%, respectively. The 17% group has the longest time for volleyball.

As shown in Table 2, when the protein nutrition level reaches 17%, the volleyball exercise time is extended. In other words, the replacement protein intake has an inhibitory effect on volleyball, but more than 17% of protein absorption does not promote the effect of volleyball. On the contrary, it will increase the burden on the body, which is counterproductive.

As shown in Figure 1, as the number of days of feeding increased, the weight distribution of rats with three protein nutritional levels increased. However, as can be seen, there is still a certain difference in weight between the 7%, 17%, and 27% groups. From the tenth day of feeding, the body weights of the three groups of rats began to differ. On the tenth day, the average weights of the three groups of rats were 92 g, 95 g, and 95 g, respectively. However, after 15 days of feeding, the average body weights of the three groups of rats were 110 g, 122 g, and 130 g, respectively, and the gap gradually widened. Overall, 7% of rats weighed slightly less than 17% and 27%, mainly because they played volleyball. Protein, sugar, and other substances are consumed during exercise, and the protein nutrition level of the 7% group obviously cannot meet the consumption demand of endurance sports such as volleyball. There was almost no difference between the 17% group and the 27% group.

### 5.2. Analysis of the Results of Nitrogen Balance Determination of Protein Metabolism in Volleyball

As shown in Figure 2, the nitrogen balance values before, during, and after volleyball in the 7% group, 17% group, and 27% group were analyzed. Due to the different levels of protein nutrition before exercise, the nitrogen balance of the three groups showed different degrees of positive nitrogen balance. The nitrogen balance data of the 17% group is in the middle. Compared with the other two groups, the nitrogen balance value of this group has a smaller degree of change. The 27% group had the highest nitrogen balance value and the degree of change was also greater. The nitrogen balance value of the 7% group was lower and showed a downward trend after volleyball, from 293 mg/day before exercise to 246 mg/day after exercise. During and after exercise, the nitrogen balance of each group changed significantly. On the third day of exercise, there was a significant difference in the positive nitrogen balance between the 7% group and the 17% group. On the fourth day of exercise, the positive nitrogen balance values of each group showed a downward trend, while the 7% group was still significantly lower than the 17% group, the 7% group was 250 mg/day, and the 17% group was 343 mg/day. On the fifth day of exercise, the nitrogen balance of the 7% group continued to decline, and a negative nitrogen balance appeared. On the second day after the rest, the nitrogen balance of group 7%, group 17%, and group 27% began to rise and returned to the preexercise state. There was no significant difference between the groups. On the 4th day after exercise, the nitrogen balance value of the 7% group fluctuated downward, which was significantly different from the 17% group and the 27% group. On the sixth day after exercise, the nitrogen balance of each group returned to the level before the experiment, and there was no significant difference between the groups. Before exercise, during, and after exercise, the nitrogen balance values of each group were different, but overall, there was no significant difference between the nitrogen balance values of the 17% group and the 27% group, which was significantly higher than that of the 7% group.

### 5.3. Analysis of the Effect of Protein Nutrition Level on Gastrocnemius Muscle Nitrogen Content and Liver Nitrogen Content during Protein Metabolism

Blood urea nitrogen (BUN) is the end product of protein metabolism, which is mainly discharged with urine through glomerular filtration. The determination of serum urea nitrogen can also be widely used as a reliable chemical indicator to measure the decomposition and metabolism of protein in the body. The increase in the content of urea nitrogen in the human blood indicates an increase in the normal catabolism of protein. Input the data of serum urea nitrogen concentration into MATLAB to establish the analysis model of serum urea nitrogen concentration of three protein nutrition levels.

As shown in Figure 3, after volleyball, the serum urea nitrogen concentrations of group 7%, group 17%, and group 27% were significantly higher than those of the control group, indicating that exercise can lead to increased protein catabolism. In volleyball, the experimental group increased the serum urea nitrogen concentration by 7%, 17%, and 27%, respectively. The difference was obvious. In volleyball, the 7% group had the largest increase in the concentration of urea nitrogen, and the 27% increase had the smallest increase, which was only 13.4%. The 27% group had a very high prevolleyball serum urea nitrogen level due to high protein intake. This level has increased before and after the experiment, but it still does not mean that the protein decomposition level of this group is low. The serum nitrogen concentration of the 17% group was elevated at a moderate level, slightly lower than that of the 7% group. This indicates that the protein nutrition level during volleyball exercise has no significant effect on the serum urea concentration in the body.

As shown in Figure 4, the first and second groups show the data of the gastrocnemius nitrogen content of the control group and the experimental group, and the fourth and fifth groups show the data of the liver nitrogen content of the control group and the experimental group. There was no significant difference in the content of gastrocnemius muscle nitrogen in the control group 7% group, 17% group, and 27% group. After volleyball, the gastrocnemius nitrous content of the three nutritional levels of the experimental group was significantly lower than that of the control group. The content of gastrocnemius in the third group was decreased in 7% group, 17% group, and 27% group. It can be seen that with the improvement of protein nutrition level, the content of gastrocnemius muscle nitrogen gradually decreases after exercise. The ability of skeletal muscles to degrade amino acids is not strong. After exercise, a large amount of muscle amino acids must be transported to the liver for metabolism. Decreased skeletal muscle nitrogen content indicates increased protein breakdown. In this experiment, it was observed that the gastrointestinal nitrogen content of all experimental groups decreased after exercise, and the gastrointestinal nitrogen content of the 7% group significantly decreased, reaching 5.2%, indicating strong protein decomposition. The reduction in gastrocnemius nitrous acid was similar in the 17% and 27% groups (4.3% and 3.6%, respectively) but less than in the 7% group.

## 6. Conclusions

Aiming at some shortcomings and shortcomings of cloud computing itself, this paper implements a data analysis system based on edge computing. Corresponding designs and implementations are made for the specific application of the algorithm under different experiments. Successfully exploring the experimental results in line with the theme of the article, the following are specific experimental data results.

1. 7% of the rats ingested the protein level required by physiology, 17% of the rats ingested the protein level of a balanced diet, and 27% of the rats ingested high protein. In the experiment, the time from volleyball to exhaustion was used to observe the effects of different protein levels on the exercise endurance of rats. The 17% group had the longest exercise time, which could be extended by 25%, and showed stronger exercise endurance, while the 27% group did not show stronger exercise endurance.
2. Nitrogen balance test is a classic method for studying protein requirements. After volleyball, the nitrogen balance of rats in each group was significantly lower than before volleyball, indicating that the decomposition and utilization of protein were enhanced. The nitrogen balance values of the 7% group and the 27% group have been changing greatly and have been showing a downward trend, and this exercise has a great influence on the nitrogen storage in the body, indicating that the intake of low protein and high protein is not conducive to the body's nitrogen storage. This experiment also observed the nitrogen content in the rat's gastrocnemius muscle and liver after volleyball. The results also show that an appropriate level of protein nutrition can help reduce the breakdown of muscle protein during exercise.
3. Therefore, proper protein content can also increase exercise endurance. Volleyball exercises cause protein breakdown in rats with low protein levels. The strongest balanced diet intake of high protein content protein is somewhat similar to that in rat protein breakdown. In addition, high protein intake will increase the burden on the human body and cause waste. Therefore, for volleyball endurance sports, a balanced dietary intake of protein quality is beneficial. That is, a protein nutrition level of 17% can promote protein metabolism during volleyball sports.

## Figures and Tables

**Figure 1:** Feeding days and weight gain in 7% group, 17% group, and 27% group.

**Figure 2:** Nitrogen balance of rats during volleyball sport with three protein nutrition levels.

**Figure 3:** Comparative analysis of the effect of protein nutrition level on serum urea nitrogen concentration.

**Figure 4:** Gastrocnemius muscle nitrogen content and liver nitrogen content of the control group and the experimental group.

**Table 1:** Feed formula with three protein nutrition levels (g/100 g).

Ingredient	Protein nutrition level		
	7%	17%	27%
Casein	8.3	20.1	31.9
Methionine	0.3	0.3	0.3
Corn starch	15.0	15.0	15.0
Sucrose	61.8	50.0	38.2

**Table 2:** Three protein nutritional levels volleyball time (minutes).

Protein nutrition level (%)	Volleyball time	Percentage (%)
7	374.2 ± 141.0	122
17	405.4 ± 154.6	125
19	400.2 ± 148.8	123
21	385.1 ± 140.8	118
27	308.2 ± 108.4	108

## Data Availability

No data were used to support this study.

## References

[1] Marcinko K., Steinberg G. R. (2015). The role of ampk in controlling metabolism and mitochondrial biogenesis during exercise. *Experimental Physiology*.

[2] Shi H., Zhu J., Luo J. (2015). Genes regulating lipid and protein metabolism are highly expressed in mammary gland of lactating dairy goats. *Functional & Integrative Genomics*.

[3] Srinivasa K. G., Sowmya Bj B. J., Shikhar A., Utkarsha R., Singh A. (2018). Data analytics assisted internet of Things towards building intelligent healthcare monitoring systems. *Journal of Organizational and End User Computing*.

[4] Maltais M. L., Perreault K., Courchesne-Loyer A. (2016). Effect of resistance training and various sources of protein supplementation on body fat mass and metabolic profile in sarcopenic overweight older adult men: a pilot study. *International Journal of Sport Nutrition and Exercise Metabolism*.

[5] Wan S., Gu Z., Ni Q. (2020). Cognitive computing and wireless communications on the edge for healthcare service robots. *Computer Communications*.

[6] Zhang X., Lu J., Li D. (2021). Confidential information protection method of commercial information physical system based on edge computing. *Neural Computing & Applications*.

[7] Mitchell W. K., Wilkinson D. J., Phillips B. E., Lund J. N., Smith K., Atherton P. J. (2017). Human skeletal muscle protein metabolism responses to amino acid nutrition. *Advances in Nutrition an International Review Journal*.

[8] Ato S., Fujita S. (2017). Regulation of muscle protein metabolism by nutrition and exercise. *The Journal of Physical Fitness and Sports Medicine*.

[9] Alghannam A.. , F., Jedrzejewski D., Bilzon J., Thompson D., Tsintzas K., Betts J.. , A. . (2016). Influence of post-exercise carbohydrate-protein ingestion on muscle glycogen metabolism in recovery and subsequent running exercise. *International Journal of Sport Nutrition and Exercise Metabolism*.

[10] Atherton P. J., Phillips B. E., Wilkinson D. J. (2015). Exercise and regulation of protein metabolism. *Progress in Molecular Biology and Translational Science*.

[11] Lalia A. Z., Dasari S., Robinson M. M. (2017). Influence of omega-3 fatty acids on skeletal muscle protein metabolism and mitochondrial bioenergetics in older adults. *Aging*.

[12] Chibisa G. E., Vinyard J. R., Laarman A. H. (2018). Short communication: effects of meloxicam administration on protein metabolism and growth performance in transported Jersey calves. *Journal of Dairy Science*.

[13] Czubowicz K., Wójtowicz S., Wencel P. L., Strosznajder R. P., Leonard P., Strosznajder R. P. (2018). The role of ceramide and sew 2871 in the transcription of enzymes involved in amyloid B precursor protein metabolism in an experimental model of alzheimer’s disease. *Folia Neuropathologica*.

[14] Meij B. S. V. D., Groot L. M. D., Deutz N. E., Engelen M. P. (2019). Effects of acute oral feeding on protein metabolism and muscle protein synthesis in people with cancer. *Nutrition*.

[15] Lv Z., Chen D., Wang Q. (2020). Diversified technologies in internet of vehicles under intelligent edge computing. *IEEE Transactions on Intelligent Transportation Systems*.

[16] Hamidi H., Jahanshahifard M. (2018). The role of the internet of Things in the improvement and expansion of business. *Journal of Organizational and End User Computing*.

[17] Wu h. h., He J., Gao y, Xue z. y (2015). Effect of protein nutrition level on protein metabolism in rats during acute exercise with different intensity. *Journal of applied medicine*.

[18] Li K. K. (2004). Research progress of exercise and protein nutrition. *Chinese Journal of Sports Medicine*.

[19] Ji-peng L., Jin-bao X., Xi-jing C., Shao-xin L. (1995). Effects of different proteins on protein and energy metabolism in exercise rats. *Chinese Journal of Nutrition*.

[20] Xin-wen C., Zhang Y.-m., Wang Z., Kong Z.-x., Su H., Yu J.-j. (2019). Effects of high-intensity interval training on the anabolism and catabolism of skeletal muscle protein in rats. *Journal of Wuhan Institute of Physical Education*.

